The article "Effect of Double-Channel Anastomosis and Esophagojejunal Anastomosis on Postoperative Recovery and Complications of Laparoscopic D2 Radical Gastrectomy for Gastric Cancer" was retracted in 2023. Reasons: signs of a paper mill; suspected computer-generated content; unreliable results or conclusions; concerns about the data.

# Effect of Double-Channel Anastomosis and Esophagojejunal Anastomosis on Postoperative Recovery and Complications of Laparoscopic D2 Radical Gastrectomy for Gastric Cancer

**DOI:** 10.1155/2022/8281558

**Published:** 2022-03-23

**Authors:** Nansheng Liao, Chaowei Xu, Shuang Zheng, Rongguo Wang

**Affiliations:** Department of General Surgery, Taizhou First People's Hospital, Taizhou 318020, China

## Abstract

The aim of this study was to investigate the effects of double-channel anastomosis versus esophagojejunostomy on postoperative recovery and complications after laparoscopic D2 radical gastrectomy for early proximal gastric cancer. The cases were collected from 100 patients with early proximal gastric cancer admitted to our hospital from January 2017 to January 2021. According to different surgical methods, they were divided into control group (total gastrectomy + esophagojejunal anastomosis) and experimental group (D2 radical resection + double-channel anastomosis). The two groups were compared in terms of clinical outcomes (operative time, intraoperative blood loss, number of lymph nodes dissected, digestive tract anastomosis time, postoperative exhaust, and hospitalization days), postoperative complications, and nutritional status; the expression of T lymphocyte subsets in peripheral blood of the two groups was detected to reflect the recovery of immune ability. There was no significant difference between the observation group and the control group in clinical operation effect indexes (*P* < 0.05). The incidence of complications of dumping syndrome and reflux esophagitis in the observation group was significantly lower than that in the control group (*P* < 0.05). In terms of postoperative nutritional status, the ratio of plasma albumin level and body weight restored to operation at 12 and 24 weeks after operation in the observation group was significantly higher than that in the control group (*P* < 0.05). 3 months after the operation, the levels of CD3 +, CD4 + cell subsets, and CD4+/CD8+ index reflecting the recovery of immune ability in the observation group were significantly higher than those in the observation group (*P* < 0.05). The application of double-channel anastomosis in laparoscopic D2 radical gastrectomy for early proximal gastric cancer has a better effect on reducing complications and promoting postoperative recovery, which is of great application value.

## 1. Introduction

Malignant gastric cancer tumors usually occurring in the upper 1/3 of the lesser curvature of the stomach, fundus of the stomach, and cardia are proximal gastric cancer. For a long time, surgery has been the only possible treatment for gastric cancer, so surgical surgery is the first choice for clinical treatment of gastric cancer. However, the surgical methods for proximal gastric cancer are still controversial abroad [1, 2]. Clinically, total gastrectomy combined with esophagojejunum Roux-EN-Y anastomosis is often performed for the surgical treatment of proximal gastric cancer, but there are many postoperative complications such as reflux esophagitis, which greatly affect the postoperative quality of life of patients [3]. With the continuous improvement of people's living standards and surgical techniques, the surgical treatment of gastric cancer should not only focus on the extension of patients' survival, but also on the improvement of patients' postoperative quality of life [4]. Therefore, proximal gastrectomy and different anastomotic methods have been explored to further improve the quality of life of patients with gastric cancer.

The article "Effect of Double-Channel Anastomosis and Esophagojejunal Anastomosis on Postoperative Recovery and Complications of Laparoscopic D2 Radical Gastrectomy for Gastric Cancer" was retracted in 2023. Reasons: signs of a paper mill; suspected computer-generated content; unreliable results or conclusions; concerns about the data.

This study investigated the effects of D2 radical gastrectomy combined with two-channel anastomosis and total gastrectomy combined with esophagojejunal anastomosis on postoperative recovery, complications, and immune recovery of patients with early laparoscopic proximal gastric cancer, in order to provide a reference for the selection of clinical proximal gastrectomy. The report was as follows.

## 2. Materials and Methods

### 2.1. Basic Information

The cases were collected from 100 patients with early proximal gastric cancer admitted to our hospital from January 2017 to January 2021 and were divided into control group and experimental group according to different surgical procedures. Among the 50 patients in the control group, 31 were female patients and 19 were male patients. The age ranged from 42 to 73 (58.66 ± 7.65) years; tumor diameter ranged from 1 to 3 (2.21 ± 1.09) cm; PT staging: 28 cases in stage 1a and 22 cases in stage 1b; PN stage 0: 20 cases, PN stage 1: 25 cases, and 2: 5 cases, respectively. Lymphatic infiltration: negative in 39 cases and positive in 11 cases. In the experimental group, there were 32 female patients and 18 male patients, respectively. The age ranged from 46 to 74 (59.20 ± 7.81) years; tumor diameter ranged from 1 to 3 (2.23 ± 1.08) cm; PT staging: 27 cases in stage 1A and 23 cases in stage 1B; PN staging: stage 0, stage 1, and stage 2: 21, 24, and 5, respectively. Lymphatic infiltration: negative in 37 cases and positive in 13 cases. There was no significant difference in general data between groups (Table 1) (*P* > 0.05).

### 2.2. Inclusion and Exclusion Criteria

Inclusion criteria were defined as follows: all patients who were in accordance with WHO Diagnostic Criteria for gastric cancer and the diagnosis was confirmed by gastroscopy, X-ray, and enhanced CT/endoscopic ultrasonography before surgery; cardia, fundus of the stomach, and upper 1/3 of the lesser curvature of the stomach; patients who can tolerate surgery without other contraindications; informed consent was signed by the patient and his family. This study was approved by the Ethics Committee of Taizhou First People's Hospital. Exclusion criteria were defined as follows: those who had undergone abdominal or other operations; patients who were accompanied by mental diseases; patients with language expression and comprehension disorders; women who are pregnant or breastfeeding; patients with serious heart, lung, liver, or kidney diseases; and patients who combined with other parts of the operation.

The article "Effect of Double-Channel Anastomosis and Esophagojejunal Anastomosis on Postoperative Recovery and Complications of Laparoscopic D2 Radical Gastrectomy for Gastric Cancer" was retracted in 2023. Reasons: signs of a paper mill; suspected computer-generated content; unreliable results or conclusions; concerns about the data.

### 2.3. Methods

Preoperative ultrasound endoscopy or enhanced CT was performed to determine the size, location, and depth of infiltration of the tumor in both groups, all by the same group of surgeons. The anesthesia method of all patients was general anesthesia with tracheal intubation, and the supine leg position was selected [5]. A small longitudinal incision was made about 1 cm below the umbilical foramen to establish pneumoperitoneum, and the pneumoperitoneum pressure was maintained at 1.6–2.0 kPa. A Trocar with a diameter of 10 mm was placed into the observation hole. A small incision was made at 1 cm below the costal margin of the left axillary front and 2 cm above the umbilicus of the midline of the left clavicle, and a Trocar with a diameter of 12 mm and 5 mm were, respectively, placed as the main and auxiliary operation holes. A small incision was made at the corresponding position on the right side, and a Trocar with a diameter of 5 mm was placed as the auxiliary operation holes of the main operation. D2 lymph node dissection was performed for early proximal gastric cancer, and lymph nodes of group No. 1, No. 2, No. 3, No. 4sa, No. 7, No. 8a, No. 9, No. 11p, No. 19, and No. 20 were sequentially dissected. Digestive tract reconstruction. (1) Observation group: double-channel anastomosis was performed. We separated the stomach while preserving the distal stomach 8–12 cm, rotated the esophagus 90° clockwise to make an incision (15 cm) from the jejunal scar of the Treitz ligament, with the navel as an adjunct, and made an incision about 3 cm around the umbilicus, fold the distal jejunum closed from the in vitro marker, proximal jejunal stump to the distal jejunum 60 cm to one side, while manually suturing the common opening and closing the mesenteric fissure. A lateral jejunal anastomosis is performed between the jejunum and the remnant gastric greater curvature 30 cm proximal to the jejunal anastomosis, and the common opening is manually sutured. The distal stump of the jejunum taken from the anterior segment of the upper colon was subjected to an esophagojejunostomy and the common opening was sutured to reconstruct the digestive tract (see Figure 1). (2) Control group: jejune-esophagus anastomosis was performed. The lower part of the esophagus was cut off at 2 cm above the cardia, the jejunum was cut off at 15 cm from the trowel's ligament, and the distal jejunum stump was sutured. End-to-end jejunum anastomosis was performed in the esophagus, and end-to-end jejunum anastomosis was performed at 45 cm from the proximal jejunum anastomosis. Finally, the mesangial foramen was closed, and the digestive tract reconstruction was completed.

The article "Effect of Double-Channel Anastomosis and Esophagojejunal Anastomosis on Postoperative Recovery and Complications of Laparoscopic D2 Radical Gastrectomy for Gastric Cancer" was retracted in 2023. Reasons: signs of a paper mill; suspected computer-generated content; unreliable results or conclusions; concerns about the data.

### 2.4. Observation Index

(1) Clinical surgical effect evaluation: indicators include surgical time, digestive tract anastomosis time, intraoperative blood loss, postoperative first exhaust time, postoperative hospital stay, etc. (2) Postoperative complications were observed; (3) Evaluation of postoperative nutritional status: the evaluation criteria were whether the plasma albumin level and body weight were restored to the preoperative level at 12 and 24 weeks after surgery. (4) The levels of T lymphocyte subsets (CD3+, CD4+, CD8+, and CD4+/CD8+) in peripheral blood were detected by flow cytometry before and 3 months after operation.

### 2.5. Statistical Analysis

Statistical Product and Service Solutions (SPSS) statistical software (version 25.0) (IBM, Armonk, NY, USA) was used for comparative analysis of the study indicators of 100 patients with early proximal gastric cancer. The comparison of counting data (complications and nutritional status assessment) was performed by *χ*^2^ test, represented by (*n*(%)); the comparison of measurement data (clinical surgical effect assessment, each immune cell index) was performed by *t*-test, represented by (‾*x* ± *s*). *P* < 0.05 indicates significant difference between groups.

## 3. Results

### 3.1. Comparison of Surgical Indicators between the Two Groups

The operative duration, digestive tract anastomosis time, lymph node dissection number, intraoperative blood loss, postoperative exhaust time, and postoperative hospitalization days in the observation group were not significantly different from those in the control group (*P* > 0.05), as shown in Table 2.

### 3.2. Postoperative Complications Were Compared between the Two Groups

There was no significant difference in the incidence of anastomotic fistula and postoperative obstruction between the two groups (*χ*^2^ = 0.315, 0.315, *P* > 0.05), but the incidence of dumping syndrome and reflux esophagitis in the observation group was significantly lower than that in the control group (*χ*^2^ = 0.046, 0.029, *P* < 0.05), as shown in Table 3.

The article "Effect of Double-Channel Anastomosis and Esophagojejunal Anastomosis on Postoperative Recovery and Complications of Laparoscopic D2 Radical Gastrectomy for Gastric Cancer" was retracted in 2023. Reasons: signs of a paper mill; suspected computer-generated content; unreliable results or conclusions; concerns about the data.

### 3.3. The Nutritional Status of the Two Groups at 3 and 6 Months after Operation Was Compared

The proportion of plasma albumin level and body weight recovered to preoperation in the observation group 12 and 24 weeks after operation was significantly higher than that in the control group (*χ*^2^ = 0.044, 0.043, 0.041, 0.045, *P* < 0.05), as shown in Table 4.

### 3.4. Comparison of Peripheral Blood T Lymphocyte Subsets between the Two Groups before and after Operation

There were no significant differences in the proportion of T lymphocyte subsets (CD3+, CD4+, CD8+) and immune index (CD4+/CD8+) between the two groups before operation (*P* > 0.05). Three months after surgery, CD3+, CD4+, and CD4+/CD8+ in peripheral blood T lymphocyte subsets of patients in the observation group were higher than those in the control group, while CD8+ was lower than those in the control group, as shown in Table 5 and Figure 2.

## 4. Discussion

At present, the surgical methods and digestive tract reconstruction methods for proximal gastric cancer are controversial [5, 6]. Although total gastrectomy (esophagojejunal anastomosis) has a wide range of resections, there is no significant difference in 3-year and 5-year survival rate between total gastrectomy and proximal gastrectomy [6, 7]. In addition, due to the destruction of the normal anatomical and physiological structure of the digestive tract and loss of duodenal access, a series of complications such as reflux esophagitis, dumping syndrome, malabsorption, weight loss, and anemia occurred in total gastrectomy [8]. Compared with total gastrectomy, proximal gastrectomy (esophagogastrostomy) retains duodenal access well and is more consistent with gastric physiological function. However, there are many postoperative complications, especially reflux esophagitis, which have a serious impact on the postoperative quality of life of patients [9].

At present, there are few studies on the recovery and complications of laparoscopic D2 radical gastrectomy for gastric cancer by double-channel anastomosis and esophagojejunostomy. Therefore, in order to further clarify the advantages and disadvantages of these two surgical methods, relevant studies were carried out. On balance, proximal gastrectomy has more advantages in postoperative diet, nutrient absorption, and weight maintenance, but it lacks an ideal gastrointestinal anastomosis method. Studies have reported that two-channel anastomosis for proximal gastrectomy can effectively prevent postoperative reflux esophagitis, and compared with total gastrectomy, postoperative nutrition status is better, complications are fewer, and postoperative recovery is more ideal [10]. In this study, there were no significant differences between the observation group and the control group in surgical-related indicators such as operation duration, digestive tract anastomosis time, number of lymph node dissection, and intraoperative blood loss, but the incidence of dumping syndrome and reflux esophagitis in the observation group was significantly lower than that in the control group (*P* < 0.05). These results suggest that there is no significant difference between double-channel anastomosis and esophagojejunal anastomosis in terms of surgical effect, but double-channel anastomosis can effectively reduce the incidence of dumping syndrome and reflux esophagitis and has a good positive effect on preventing recurrence, which is basically consistent with the results of other scholars [11].

The article "Effect of Double-Channel Anastomosis and Esophagojejunal Anastomosis on Postoperative Recovery and Complications of Laparoscopic D2 Radical Gastrectomy for Gastric Cancer" was retracted in 2023. Reasons: signs of a paper mill; suspected computer-generated content; unreliable results or conclusions; concerns about the data.

Reconstruction of the digestive tract is very important for the recovery of gastrointestinal physiological function and motor ability. The reconstructed digestive tract should not only have a certain food storage space so that chyme can pass through the duodenum but also have the basic function of preventing reflux [12]. The principle of dual-channel match method for distal jejunum, respectively, with proximal jejunum anastomosis of the esophagus, stomach, digestive channel formation, food through esophagus jejunum anastomosis after, respectively, into the distal gastric cavity and is entered into the jejunum anastomotic 3, while other food can be directly into the small intestine, so that the first and second anastomosis can effectively prevent gastric acid reflux. In the process of food entering the distal stomach, the original function of the gastroduodenal digestive tract is retained [13]. Therefore, the incidence of dumping syndrome and reflux esophagitis in two-channel anastomosis is lower than that in total gastrectomy (esophagojejunal anastomosis). In addition, the proportion of plasma albumin level and body weight recovered to operation in the observation group was significantly higher than that in the control group at 3 and 6 months after surgery (*P* < 0.05), suggesting that two-channel anastomosis has a positive effect on improving the nutritional status and quality of life of patients after surgery. From the perspective of radical treatment, total gastrectomy is not necessary for middle stomach (U zone) cancer, while proximal gastrectomy is the most appropriate operation, and the scope of intraoperative resection and resection is more reasonable. In addition, preserving the pylorus and duodenum through two-channel anastomosis is also conducive to food retention and mixing, promoting intestinal digestion, preventing the delayed secretion of gastrin and secretin, preventing disorder or weakening of absorption function, and thus improving the postoperative nutritional status of patients [14]. Total gastrectomy makes the stomach of patients no longer grind and decompose the food, and the fat in the food is not fully emulsified, which greatly reduces the absorption of nutrients in the intestinal tract. Patients are prone to malnutrition and significant weight loss, which leads to poor postoperative recovery or even life-threatening.

The article "Effect of Double-Channel Anastomosis and Esophagojejunal Anastomosis on Postoperative Recovery and Complications of Laparoscopic D2 Radical Gastrectomy for Gastric Cancer" was retracted in 2023. Reasons: signs of a paper mill; suspected computer-generated content; unreliable results or conclusions; concerns about the data.

At the same time, this study found that the levels of CD3+, CD4+, and CD4+/CD8+ index in peripheral blood of the observation group treated with double-channel anastomosis for early proximal gastric cancer were significantly higher than those of the control group treated with jejune-esophageal anastomosis, indicating that the recovery of immune capacity in the observation group was stronger than that in the control group. This change may be closely related to the improvement of patients' quality of life by double-channel anastomosis.

Of course, since this study was a single-center randomized controlled study, with only 50 cases in each group and a short follow-up time, more cases need to be accumulated in the future to observe and evaluate the long-term effects of two-channel anastomosis.

## 5. Conclusions

In conclusion, the application of two-channel anastomosis in laparoscopic D2 radical gastrectomy for early proximal gastric cancer has achieved satisfactory results with a low incidence of postoperative complications, effectively improving the postoperative nutritional status of patients and promoting their postoperative recovery. Therefore, it is recommended to be popularized and applied. [15].

## Figures and Tables

**Figure 1:** Operation of patients with early proximal gastric cancer treated by double-channel anastomosis.

**Figure 2:** Flow cytometry was used to detect the changes of T lymphocyte subsets in peripheral blood of 2 groups before and after operation.

**Table 1:** General data between groups.

	Observation group (*n* = 50)	Control group (*n* = 50)	t/*χ*^2^	*P*
Age (years)	59.20 ± 7.81	58.66 ± 7.65	0.349	0.726
Gender (male)	18	19	3.313	0.068
Tumor diameter (cm)	2.23 ± 1.08	2.21 ± 1.09	0.092	0.927
PT staging				
Stage 1a	27	28	0.490	0.484
Stage 1b	23	22		
PN stage				
0	21	20	0.045	0.977
1	24	25		
2	5	5		
Lymphatic infiltration				
Negative	37	39	13	0.486
Positive	13	11		

**Table 2:** Comparison of surgical indicators between the two groups (‾*x* ± *s*).

Group	*n*	The operation time (min)	Anastomosis timing (min)	Number of dissected lymph nodes (n)	Intraoperative blood loss (ml)	Postoperative exhaust time (h)	Postoperative hospital stay (d)
Observation group	50	74.83 ± 9.82	32.36 ± 7.92	35.05 ± 3.54	227.58 ± 15.38	2.17 ± 0.75	7.98 ± 0.76
Control group	50	76.32 ± 16.63	34.33 ± 5.65	34.09 ± 4.07	231.07 ± 13.38	2.26 ± 0.65	8.23 ± 0.94
*t*	—	0.546	1.432	1.258	1.211	0.641	1.462
*P*	—	0.587	0.155	0.211	0.229	0.523	0.147

The article "Effect of Double-Channel Anastomosis and Esophagojejunal Anastomosis on Postoperative Recovery and Complications of Laparoscopic D2 Radical Gastrectomy for Gastric Cancer" was retracted in 2023. Reasons: signs of a paper mill; suspected computer-generated content; unreliable results or conclusions; concerns about the data.

**Table 3:** Comparison of postoperative complications between the two groups (*n*, (%)).

Group	*n*	Anastomotic fistula	Postoperative obstruction	Dumping syndrome	Reflux esophagitis
Observation group	50	0(0.00)	0(0.00)	2(4.00)	4(8.00)
Control group	50	1(2.00)	1(2.00)	8(16.00)	12(24.00)
*χ*2	—	1.010	1.010	4.000	4.762
*P*	—	0.315	0.315	0.046	0.029

**Table 4:** The nutritional status of the two groups at 3 and 6 months after operation was compared.

Group	*n*	The plasma albumin level returned to preoperative		Weight regain to preoperative level	
		At 12 weeks postoperatively	At 24 weeks postoperatively	At 12 weeks postoperatively	At 24 weeks postoperatively
Observation group	50	32(64.00)	41(82.00)	25(50.00)	34(68.00)
Control group	50	22(44.00)	32(64.00)	15(30.00)	21(42.00)
*χ* ^2^	—	4.026	4.110	4.167	4.006
*P*	—	0.044	0.043	0.041	0.045

**Table 5:** Comparison of peripheral blood T lymphocyte subsets between the two groups before and after operation (‾*x* ± *s*).

Group	*n*	Preoperative				3 months postoperative			
		CD3+	CD4+/CD3+	CD8+/CD3+	CD4+/CD8+	CD3+	CD4+/CD3+	CD8+/CD3+	CD4+/CD8+
Observation group	50	56.63 ± 5.27	36.25 ± 4.25	57.27 ± 5.36	0.65 ± 0.15	70.65 ± 5.83	57.43 ± 4.52	37.45 ± 3.57	1.52 ± 0.12
Control group	50	55.28 ± 6.11	35.64 ± 4.75	60.24 ± 5.89	0.59 ± 0.16	62.45 ± 5.57	48.24 ± 4.11	42.14 ± 4.26	1.15 ± 0.16
*t*	—	0.194	0.246	0.893	0.257	5.357	4.854	5.986	4.986
*P*	—	0.125	0.314	1.032	0.386	0.015	0.018	0.012	0.022

## Data Availability

The datasets used and analyzed during the current study are available from the corresponding author on reasonable request.
